This article has been retracted.

# Serum amyloid a induces M2b-like macrophage polarization during liver inflammation

**DOI:** 10.18632/oncotarget.22652

**Published:** 2017-11-23

**Authors:** Yibin Wang, Haijun Huang, Renhua Sun, Bingyu Chen, Fang Han, Qian Li, Yin Ni, Xi Li, Jingquan Liu, Xiaozhou Mou, Yuexing Tu

**Affiliations:** ^1^ Department of Cardiology, Chunan First People’s Hospital, Hangzhou 311700, China; ^2^ Department of Infectious Diseases, Zhejiang Provincial People’s Hospital, People’s Hospital of Hangzhou Medical College, Hangzhou 310014, China; ^3^ ICU Department, Zhejiang Provincial People’s Hospital, People’s Hospital of Hangzhou Medical College, Hangzhou 310014, China; ^4^ Centre of Laboratory Medicine, Chunan First People’s Hospital, Hangzhou 311700, China; ^5^ Department of Transfusion Medicine, Zhejiang Provincial People’s Hospital, People’s Hospital of Hangzhou Medical College, Hangzhou 310014, China; ^6^ Centre of Laboratory Medicine, Zhejiang Provincial People’s Hospital, People’s Hospital of Hangzhou Medical College, Hangzhou 310014, China; ^7^ Clinical Research Institute, Zhejiang Provincial People’s Hospital, People’s Hospital of Hangzhou Medicine College, Hangzhou 310014, China; ^8^ Key Laboratory of Tumor Molecular Diagnosis and Individualized Medicine of Zhejiang Province, Hangzhou 310014, China

**Keywords:** serum amyloid A (SAA), liver fibrogenesis, macrophage polarization

## Abstract

Hepatitis causes hepatic cell injury, regeneration and different levels of fibrogenesis, and severe liver fibrogenesis progresses into cirrhosis with liver dysfunction. Serum amyloid A (SAA) is an acute phase protein that is predominantly secreted by hepatocytes during early injury or infection. Nevertheless, the relationship of SAA and development of cirrhosis as well as the underlying molecular mechanisms is largely unknown. Here, we found that macrophages are the major SAA-binding cells in the injured liver. *in vitro*, macrophages treated with SAA exhibited high production of IL-10 but low production of IL-12, as features for M2 macrophages. Moreover, these polarized M2 macrophages by SAA also produced IL-1, IL-6 and TNFa, characteristics for an M2b subtype, rather than an alternative M2a or fibrogenic M2c subtype. In a mouse model of carbon tetrachloride (CCl_4_)-induced hepatic fibrogenesis/cirrhosis, anti-SAA sera were used to block the effects of SAA, resulting in increases in the severity of hepatic fibrosis, suggesting an overall anti-fibrogenic effect of SAA. Isolated macrophages from mouse liver showed that anti-SAA appeared to alter the polarization of macrophages from M2b to M2c, suggesting that SAA may induce M2b-like macrophage polarization during liver inflammation, which prevents the liver from fibrogenesis.

## INTRODUCTION

An inflammation of the liver causes hepatitis, among which hepatitis C infection is known to be the leading cause of chronic liver disease, cirrhosis and hepatocellular carcinoma [1]. The pathology of cirrhosis is characterized with chronic hepatic inflammation, portal hypertension, and disruption of normal hepatic architecture [1]. Carbon tetrachloride (CCl_4_) intraperitoneal injection has been widely used to generate an animal model for studying liver fibrogenesis and cirrhosis in humans [2]. Despite of recent advances in dissecting the molecular regulation in the control of cirrhosis development after liver infection, our understanding of this prevalent disease remains limited.

Serum amyloid A (SAA) is a 12.5 kd acute phase protein which play a regulatory role during inflammation [3]. After infection or injury, SAA levels may increase up to 1000-fold in serum, and SAA is typically found in association with high density lipoproteins (HDL) in circulation [3]. Previous studies have shown that SAA is predominantly produced and secreted by hepatocytes, after stimulated by LPS and TNFα in a NF-κB dependent manner [4]. Many studies have demonstrated a role of SAA in inflammatory diseases such as atherosclerosis [5] and rheumatoid arthritis [4], seemingly through control of different signaling pathways including NF-κB, JNK, C/EBP, JNK, Erk/MAPK and PI3k/Akt/mTor [6]. However, the effects of SAA on liver inflammation and fibrogenesis remain poorly defined.

Macrophages processes a number of different receptors for lineage-determining growth factors, T helper (Th) cell cytokines, etc [7]. Macrophages mature in tissue and are activated in a dynamic response to environmental stimuli to acquire specialized functional phenotypes as classic vs. alternative, also M1 (high production of interleukin-12 (IL-12) and low production of IL-10) and M2 (high production of IL-10 and low production of IL-12), respectively [8]. However, the complex activation of M2 macrophages renders the dichotomy for them into M2a, M2b and M2c categories [9]. The common denominator of 3 M2 subpopulations is high IL-10 production accompanied by low production of IL-12 [9]. Another pan M2 signature is their production of enzyme Arginase-1 that depletes L-arginine in competition with iNOS for substrate [9]. M2a macrophages are CD163-high, CD206-high, but negative for IL-1, IL-6, tumor necrosis factor (TNFa) and transforming growth factor beta (TGFb), M2b macrophages are negative for CD163, CD206 and TGFb, but expressed high levels of IL-1, IL-6 and TNFa, and M2c macrophages are CD163-high, CD206-high, and expressed high TGFb, but negative for IL-1, IL-6, TNFa [9]. Among the subtypes of M2 macrophages, M2c is highly fibrogenic, compared to M2a and M2b [9]. Of note, SAA appeared to control a variety of cytokines and chemokines, many of which play critical roles in the macrophage differentiation and polarization [6]. Thus, it is expected that many of the functions of SAA may be conducted through its effects on macrophages. However, the effects of SAA on macrophage polarization during liver inflammation and fibrogenesis are largely unknown. Here we addressed this question.

We found that macrophages are the major SAA-binding cells in the injured liver. *in vitro*, macrophages treated with SAA appeared to polarize to an M2b subtype, rather than an M2a or fibrogenic M2c subtype. In a mouse model of CCl_4_-induced hepatic fibrogenesis/cirrhosis, anti-SAA sera blocked the effects of SAA, resulting in increases in the severity of hepatic fibrosis, suggesting an overall anti-fibrogenic effect of SAA, which was further supported by the fact that anti-SAA altered the polarization of macrophages from an M2b to a fibrogenic M2c subtype.

## RESULTS

### Macrophages are the major SAA-binding cells in the injured liver

Carbon tetrachloride (CCl_4_) was used to treat mice for 8 weeks, after which the mouse liver was stained for F4/80, a pan-macrophage marker (Figure 1A), and for SAA (Figure 1B). Interestingly, the signals from F4/80+ macrophages and from SAA in the mouse liver appeared to very similar from immunohistochemistry images (Figure 1A-1B), suggesting that macrophages may be a major SAA-binding cells in the injured liver. To prove this hypothesis, we dissociated CCl_4_-treated mouse liver into signal cells, and analyzed expression of SAA and F4/80 on the surface of these cells by flow cytometry. We found that about half of the SAA+ cells (represent SAA-binding cells) were F4/80+, suggesting that macrophages represent half of the total SAA-binding cells in the injured liver (Figure 1C). On the other hand, most of F4/80+ cells appeared to be SAA+, suggesting that most of the macrophages bind to SAA in the injured liver (Figure 1C). Moreover, significantly lower levels of SAA mRNA were detected in purified F4/80+ macrophages, compared to F4/80- non-macrophage cells (Figure 1D), suggesting that SAA was not predominantly produced by macrophages, consistent with previous reports showing that hepatocytes are major SAA-producing cells in the injured liver. Indeed, SAA+F4/80- cells appeared to be the relative small population of cells in liver that SAA attached to, and these cells seemed to be mainly endothelial cells. On the other hand, SAA-/F4/80- cells should be mainly hepatocytes. Thus, macrophages are the major SAA-binding cells in the injured liver.

**Figure 1:** Macrophages are the major SAA-binding cells in the injured liver **(A-B)** Immunohistochemistry for F4/80 (A) and SAA (B) in mouse liver 8 weeks after carbon tetrachloride (CCl_4_) treatment. **(C)** Representative flow chart for F4/80 and SAA in dissociated mouse liver 8 weeks after CCl_4_ treatment. **(D)** RT-qPCR for SAA mRNA in purified F4/80+ vs F4/80- cells from dissociated mouse liver 8 weeks after CCl_4_ treatment. *p<0.05. n=5. Scale bars are 50 μm.

### SAA induces M2b macrophage polarization *in vitro*

In order to understand the effects of SAA binding on macrophage differentiation and polarization, we treated cultured bone marrow derived macrophages from untreated naive mice with SAA. Compared to non-SAA-treated macrophages (SAA-), SAA-treated macrophages (SAA+) significantly increased IL-10 production (Figure 2A), did not increase IL-12 production (Figure 2B), suggesting that SAA induces an M2-like polarization *in vitro*. Moreover, compared to non-SAA-treated macrophages, SAA-treated macrophages did not increase TGFb production (Figure 2C), suggesting that the polarized M2 macrophages were not M2c. In addition, compared to non-SAA-treated macrophages, SAA-treated macrophages significantly increased IL-1 production (Figure 2D), IL-6 production (Figure 2E), TNFa production (Figure 2F), and significantly increased CD86 expression on the cell surface (Figure 2G), but did not induce CD163 expression on the cell surface (Figure 2H), suggesting that SAA induces M2b macrophage polarization *in vitro*.

**Figure 2:** SAA induces M2b macrophage polarization *in vitro* Cultured bone marrow derived macrophages were isolated from untreated naive mice, and then treated with SAA (SAA+) or not (SAA-) for 24 hours before analysis. **(A)** ELISA for IL-10 production. **(B)** ELISA for IL-12 production. **(C)** ELISA for TGFb production. **(D)** ELISA for IL-1 production. **(E)** ELISA for IL-6 production. **(F)** ELISA for TNFa production. **(G-H)** Representative flow chart for CD86 (G), and for CD163 (H). ^*^p<0.05. NS: non-significant. n=5.

### Suppression of SAA in CCl_4_-treated mouse liver

Next, we examined the effects of SAA on liver fibrogenesis after liver injury *in vivo*. CCl_4_ was injected to induce liver injury and fibrosis in mice. Antisera of SAA were given to some mice that received CCl_4_ in order to evaluate the effects of SAA as a loss-of-function experiment. After 8 weeks, the mice were analyzed (Figure 3A). At analysis, the SAA levels were first quantified in the mouse liver to confirm the interference with SAA activity by antisera of SAA. We found that SAA levels in mouse liver were significantly increased by CCl_4_, but this increase in SAA was significantly attenuated by antisera of SAA (Figure 3B). Moreover, the histology of mouse liver showed that the severe morphological changes in CCl_4_-treated mouse liver seemed to aggravate by using antisera of SAA (Figure 3C).

**Figure 3:** Suppression of SAA in CCl_4_-treated mouse liver **(A)** CCl_4_ was injected to induce liver injury and fibrosis in mice. Antisera of SAA were given to some mice that received CCl_4_ in order to evaluate the effects of SAA as a loss-of-function experiment. After 8 weeks, the mice were analyzed. **(B)** At analysis, the SAA levels were quantified by RT-qPCR in the mouse liver. **(C)** Representative histology of mouse liver. ^*^p<0.05. n=10. Scale bars are 50 μm.

### Suppression of SAA enhances liver fibrogenesis induced by CCl_4_

Then we quantified the changes in liver fibrosis and function. We found that antisera of SAA further augmented the increases in the percentage of the fibrotic area by CCl_4_ (Figure 4A). For assessment of liver function, portal hypertension and sodium metabolism were analyzed, showing that antisera of SAA further increased the portal pressure (Figure 4B), and sodium balance (Figure 4C) by CCl_4_, probably through a reduced sodium excretion (Figure 4D). These data suggest that suppression of SAA enhances liver fibrogenesis induced by CCl_4._

**Figure 4:** Suppression of SAA enhances liver fibrogenesis induced by CCl_4_ **(A)** The fibrotic area at sacrifice was evaluated after Sirius red staining, shown by the percentage of the fibrotic area. **(B)** Portal pressure. **(C)** Sodium balance. **(D)** Sodium excretion. ^*^p<0.05. n=10.

### Antisera of SAA alters the polarization of macrophages from M2b to M2c in the injured liver

For determining the underlying mechanisms, we Isolated macrophages from mouse liver (Figure 5A) and analyzed the levels of cytokines and expression of surface markers related to macrophage subtype categories, based on our *in vitro* results. We found that anti-SAA did not alter the increased IL-10 production by SAA (Figure 5B), did not increase IL-12 production (Figure 5C), suggesting that SAA suppression did not induce a polarization between M1 and M2 macrophages in the injured mouse liver. Moreover, anti-SAA significantly increased TGFb production (Figure 5D), suggesting that SAA suppression may favor M2c polarization. Since M2c is known to be highly fibrogenic, these data explained the increased in liver fibrogenesis and dysfunction by SAA suppression in the injured moues liver (Figure 4A-4D). In addition, anti-SAA appeared to attenuate the production of IL-1 (Figure 5E), IL-6 (Figure 5F), and TNFa (Figure 5G), and to attenuate the increases in CD86 expression on the cell surface by CCl_4_ (Figure 5H), consistent with a reduction in M2b macrophages and an increase in M2c macrophages. Furthermore, anti-SAA induced the surface expression of CD163 on macrophages from CCl_4_-treated mouse liver (Figure 5I), also consistent with a reduction in M2b macrophages and an increase in M2c macrophages. Together, these data suggest that SAA suppression may alter the polarization of macrophages from M2b to M2c in the injured mouse liver, or SAA may induce M2b-like macrophage polarization and prevents M2c-like macrophage polarization during liver inflammation, which prevents the liver from fibrogenesis.

**Figure 5:** Antisera of SAA alters the polarization of macrophages from M2b to M2c in the injured liver **(A)** Macrophages were isolated from mouse liver by flow cytometry. **(B)** ELISA for IL-10 production. **(C)** ELISA for IL-12 production. **(D)** ELISA for TGFb production. **(E)** ELISA for IL-1 production. **(F)** ELISA for IL-6 production. **(G)** ELISA for TNFa production. **(H-I)** Representative flow chart for CD86 (H), and for CD163 (I). ^*^p<0.05. NS: non-significant. n=10.

## DISCUSSION

More than 20 years ago, it was discovered that IL-4 and interferon-gamma (IFNr) or lipopolysaccharide (LPS) induced different macrophage gene expression profile [10]. While IFNr-activated macrophages are termed classical activated macrophages, or M1 macrophages, IL-4-activated macrophages are termed alternative activated macrophages, or M2 macrophages, according to the differential macrophage arginine metabolism in various mouse strains with T helper type 1 and T helper type 2 backgrounds [10]. In 2004, Mantovani et al. further divided M2 macrophages into M2a, M2b and M2c subtypes based on the applied stimuli and the induced transcriptional changes [11]. Nowadays, the M1/M2 (subtypes) classification of macrophages is found to be an oversimplified criteria since the spectrum of macrophage populations appear to be far more diverse and complex [12].

In the current study, we used female mice to investigate the macrophage polarization induced by SAA during liver injury, since we found that CCl_4_ induced hepatic cirrhosis more consistently in female mice. SAA is primarily produced and secreted by hepatocytes, and released into circulation where SAA is predominantly associated with HDL but locally SAA seemed to bind to macrophages and some other cells other than hepatocytes [3]. Indeed, it has been reported that hepatic stellate cells (HSCs) are SAA-binding cells in liver [13]. Since HSCs are essential players in the liver fibrosis [14-17], it is thus speculated that SAA may play a role in liver fibrogenesis. In the current study, we showed that another SAA-binding cell type in the injured liver is macrophage. Since we found that very few macrophages in the injured liver were not attached to SAA, it seemed that both M1 and M2 macrophages should be bound by SAA. Thus, the control of macrophages by SAA may be consistent, which leads to a sustained changes in the macrophage phenotype or polarization.

Here, we used accepted criteria to determine the subtype of macrophages. First of all, the production of IL-10 and IL-12 was used to decide the M1/M2 on the top of any M2 subtypes [8]. SAA increased IL-10 but did not increase IL-12 *in vitro* and *in vivo*, suggesting that the macrophages are polarized to M2 direction by SAA. Suppression of SAA *in vivo* did not alter these IL-10/IL-12 production, which indicates that SAA should not regulate M1 vs M2 polarization.

IL-1, IL-6, TNFa and CD86 are produced by M1 and M2b macrophages, but not by M2a and M2c macrophages. On the other hand, CD163 is expressed by M2a and M2c macrophages, but not by M1 and M2b macrophages. TGFb appears to be exclusively produced by M2c macrophages [8]. Here, SAA induced IL-1, IL-6, TNFa and CD86, but not TGFb and CD163, on macrophages on the top of high IL-10 and low IL-12, which fits perfectly to the characteristics for M2b macrophage, suggesting that SAA induces M2b macrophage polarization. Interestingly, suppression of SAA *in vivo* reduced IL-1, IL-6, TNFa and CD86, but increased CD163 and TGFb, which indicates that loss of SAA shifts the polarization of M2b to M2c. The reduction but not completely loss of IL-1, IL-6, TNFa and CD86 may result from incomplete polarization of M2b to M2c and the remaining M2b contributes to these signals.

To the best of our knowledge, it is the first study to demonstrate a role of SAA in controlling macrophage polarization in injured liver. This specific effects of SAA on macrophages seemed to have a protective role against fibrosis, which may contradict the effects of SAA on HSCs in a complex regulatory network to regulate liver regeneration and function.

## MATERIALS AND METHODS

### Experimental protocol approval

All the experimental methods in the current study have been approved by the research committee at Zhejiang Provincial People’s Hospital of People’s Hospital of Hangzhou Medical College. All mouse experiments were approved by the Institutional Animal Care and Use Committee at Zhejiang Provincial People’s Hospital of People’s Hospital of Hangzhou Medical College.

### Animal manipulations

Liver injury and fibrosis were induced in female C57BL/6 mice (SLAC Laboratory Animal Co. Ltd, Shanghai, China) of 12 weeks of age by CCl_4_ intraperitoneal injection [CCl_4_ solution of 50% (v/v) in paraffin oil (Sigma-Aldrich, St. Louis, MO, USA)] at a dose of 2ml/kg body weight and frequency of twice per week for 8 weeks (CCl_4_). Control mice received intraperitoneal injection of paraffin oil of same volume and frequency (CTL). For SAA suppression, anti-SAA sera (Thermo Fisher Scientific, Shanghai, China) of 100μg were injected intraperitoneally at the same time of each CCl_4_ injection.

### *In vitro* treatment of macrophages by SAA

Primary mouse macrophages were isolated from bone marrow of female C57BL/6 mice at 12 weeks of ago, as described before [18]. Marrow was flushed out with PBS through a 23-gauge needle. Cells were pre-treated with APC-conjugated F4/80 antibody (Becton-Dickinson Biosciences, San Jose, CA, USA) and then sorted for APC+ cells by flow cytometry. Purified F4/80+ macrophages were cultured in Dulbecco’s Modified Eagle Medium (DMEM; Invitrogen, St. Louis, MO, USA) suppled with 10% fetal calf serum and 1% L-glutamine (Invitrogen). For SAA treatment, cultured macrophages were treated with recombinant mouse SAA (R&D Systems, Shanghai, China) at a concentration of 0.5 μmol/l for 24 hours before analysis.

### Flow cytometry

The antibodies used in flow cytometry were APC-conjugated anti-F4/80, PE-cy7-conjugated anti-SAA, FITC-conjugated anti-CD86 and PE-conjugated anti-CD163 (Becton-Dickinson Biosciences). Data were analyzed using FlowJo software (Flowjo LLC, Ashland, OR, USA).

### Histology and immunohistochemistry

Immunohistochemistry on mouse liver sections was performed routinely using a rabbit-anti-mouse SAA (Abcam, St. Louis, MO, USA), or a rat-anti-mouse F4/80 antibody (Becton-Dickinson Biosciences) and the signals were detected by an ABC method (Dako, Shanghai, China). H&E staining was done routinely.

### RT-qPCR

Total RNA was extracted using TRIZOL reagent (Invitrogen, shanghai, China) according to the manufacturer’s instructions. A High Capacity cDNA Reverse Transcription Kit (Applied Biosystems, Shanghai, China) was used to convert RNA into cDNA. Real-time PCR was conducted in an ABI7500 real-time PCR instrument (Applied Biosystems) with the SYBR Premix Ex Taq (Qiagen, Shanghai, China). Primers were ordered from Qiagen. A 2^-ΔΔCt^ method was used for quantification of gene expression levels. Relative expression levels of genes were obtained through sequential normalization of the values against GAPDH and experimental controls.

### ELISA

ELISA for IL-10, IL-12, IL-6, IL-1, TNFa and TGFb was performed using corresponding ELISA kits (R&D Biosystems).

### Evaluation of liver fibrosis

Mouse liver was fixed in 10% phosphate-buffered formalin, embedded in paraffin, and stained for collagen using Sirius red assay. Positive fibrotic areas were counted based on 200 random selected fields that were estimated to represent tissue of 6mm^2^ [14]. The percentage of fibrotic area was expressed as number of fibrotic fields divided by total fields, and then multiplied by 100.

### Sodium balance

The urine sodium concentration (UNa) was assayed by flame photometry (Roika 2000, Roika, UK), and renal sodium excretion (UNaV) was calculated with the following formula: UNaV = UV × UNa, where UV is urine volume. The intake of sodium was assessed by measuring the amounts of food and water consumed. Sodium balance was calculated as (Na+ provided by food and water)-UNaV.

### Portal pressure

After evaluation of sodium metabolism, under anesthesia, a PE-50 polyvinyl catheter was placed in the cecal vein. The other end of the catheter was connected to a highly sensitive transducer (ADInstruments Shanghai Trading Co. Shanghai, China) to assess portal pressure.

### Statistical analysis

The statistical analysis was performed with the GraphPad Prism 6 (GraphPad Software, San Diego, CA, USA). Comparison of 2 groups was carried out with Student’s T test. All values represent the mean ± standard deviation (SD). A value of *p*<0.05 was considered as significant. Patients’ 5-year survival was recorded by Kaplan-Meier curve.
